The article "Environmental threat in France: Two studies testing the effect of threatening messages on system justification and environmental denial" was published in 2022. Journal: Front Psychol.

# Environmental threat in France: Two studies testing the effect of threatening messages on system justification and environmental denial

**DOI:** 10.3389/fpsyg.2022.891329

**Published:** 2022-07-19

**Authors:** Hélène Labarre, Marie-Line Felonneau

**Affiliations:** Laboratoire de psychologie EA4139, Université de Bordeaux, Bordeaux, France

**Keywords:** environmental threat, system justification, environmental denial, political orientation, system threat

## Abstract

Climate change consequences are affecting our entire political, economic and social system. At a psychological level, it represents a large number of threatening events that we have to deal with. In the scientific literature, there is an active debate about the inconsistent effects of environmental threatening messages. One explanation for this inconsistency is that people respond differently to a threat, depending on some psychological dispositions. Indeed, studies on system justification theory showed that when people with a right political orientation are exposed to a threat to their system, they show a motivation to defend it. Although those tendencies have been linked to environmental denial, there is a lack of experimental studies testing the direct effect of environmental threat, especially in European context. We address this issue with two experiments in which we highlighted the environmental threat for one’s system (Study 1, *N* = 144) and for the continuity of one’s habits (Study 2, *N* = 148) in a French sample. The design was the same for both studies: three types of video-clips were presented to participants (i.e., control, neutral and threat) and we measured general system justification, environmental denial and political orientation. Our results showed no significant effect of our threat manipulation in both studies. However, they support that a right political orientation in France positively predicts system justification tendencies in study 1 and environmental denial in study 2. Findings are discussed through theoretical and methodological implications.

## Introduction

Climate change consequences are affecting not only our physical environment but also our psychological and social environment. Accordingly, it represents a multi-level threat that we have to deal with. Even though the main consequences are now irreversible (Intergovernmental Panel on Climate Change [IPCC] et al., 2021), we can still limit the severity of some disasters. To address this challenge, psychologists can help to improve the understanding of psychological and contextual barriers that undermine environmental actions (e.g., Gifford, 2011; Swim et al., 2011; Hornsey and Fielding, 2020). In this research, we will focus on the obstacle resulting from the tendency to justify one’s system and to deny environmental problems in the context of environmental threat. More specifically, we address the hypothesis proposed by Feygina et al. (2010) about the effect of the environmental threat on system justification tendencies and denial, depending on political orientation.

## Environmental threat

When authors used the expression “environmental threat” in the literature, it implicitly refers to all the negative physical, social and psychological impacts of climate change (Reser et al., 2011). The set of negative consequences referred to, in the literature, includes a large variety of phenomena that are more or less severe, more or less likely and more or less controllable. For a better understanding of its effects at the psychological level, we must first establish the perimeter of what is considered a threat. In this article, we follow the distinction by Crawford (2017) on “meaning threats” and “physical threats.” He defines physical threat as a physical danger that poses a risk to people’s safety (i.e., potential death) and meaning threat as an event that violates “one’s senses of belonging, identity, purpose, significance, continuity, or certainty” (Crawford, 2017, p. 356). Due to the numerous consequences of climate change, researchers can induce environmental threat with both types depending on their objectives. In this research, we chose to study the “general meaning threat” posed by climate change because most people in Europe have not experienced severe climate danger as described by “physical threat.” Moreover, even the meaning threat can refer to different types of threat. In this research, we decided to distinguish two levels of this general meaning threat: one concerning the political, economic and social system and the other directly concerning the continuity of individual life habits.

If most European countries are, for now, relatively spared by climate change consequences, the experience of the environmental crisis is mostly indirect through social media, newspapers or technologies (Reser et al., 2011). It is therefore common for researchers to use these same communication methods as materials to recall the threatening aspects of climate change. More specifically, inducing a sense of threat often consists of exposing people to pessimistic messages about the severity of climate change consequences. However, this type of operationalization has led to inconsistent outcomes (e.g., van Zomeren et al., 2010). On the one hand, some studies found that the perceived threat of climate change can be positively associated with personal efficacy (Byrne and Hart, 2009; Hornsey et al., 2015). Moreover, results have shown that when people are threatened by dire messages, they increase their intentions to reduce energy consumption (Hartmann et al., 2014) and engage in more pro-environmental behaviors (Kim et al., 2013). On the other hand, researchers have also found that dire messages can encourage people to deny the problem and ignore it (Feinberg and Willer, 2011; Hart and Feldman, 2014). Moreover, some studies failed to find an increase of pro-environmental intentions and behaviors (O’Neill and Nicholson-Cole, 2009; Weinstein et al., 2015). To explain these inconsistent findings, some authors found that dispositional factors, such as political orientation, may moderate individual response to threatening communication (e.g., Häkkinen and Akrami, 2014; Hoffarth and Hodson, 2016; Clarke et al., 2019). This literature is consistent with the hypothesis that, in the face of threatening climate events, people would engage in defensive cognitive processes and minimize climate change severity. It is from this perspective that this research is conducted. Among the many processes and dispositional factors that have been identified as barriers to attitudinal and behavioral changes, we focus here on system justification tendencies and political orientation (e.g., Gifford, 2011; Hornsey and Fielding, 2020).

## System justification

System Justification Theory suggests that people are motivated to enhance the legitimacy of their own system (Jost et al., 2004). A large body of research demonstrated that system justification is especially prevalent in threatening contexts and for right political ideologies (e.g., Kay and Friesen, 2011; Friesen et al., 2019; Jost, 2019). According to Jost et al. (2010), the tendency to justify one’s system is enhanced when the system is threatened or criticized. Although this effect has been shown for different types of threats (for a review, see Kay and Friesen, 2011), this claim has not yet been tested for environmental threat. According to Feygina et al. (2010), climate change can be considered as a threat to the system because acknowledging the role of human activity would imply challenging the foundations of our social, political and economic system. Indeed, climate change represents, *per se*, a threat to the significance of the current system and to the continuity of individuals’ habits. It has been proposed that system justification tendencies and environmental denial can be increased by environmental threat, specifically for right political orientation but, to our knowledge, there are only few studies that investigate this issue (e.g., Clarke et al., 2019). Testing this effect is the first objective of this research.

In the United States political system there is strong evidence that right political orientation and conservatism are positively associated with system justification tendencies (Jost, 2019) and environmental denial (e.g., McCright and Dunlap, 2011). Several studies also demonstrated that perceived threat, system justification tendencies and right political orientation are relevant factors to understand environmental attitudes (e.g., Feygina et al., 2010; Jylhä and Akrami, 2015; Clarke et al., 2019). Moreover, a recent meta-analysis showed that political orientation and voting behavior are strong predictors of environmental denial while controlling for other sociodemographic factors (Hornsey et al., 2016). It is therefore relevant to explore the role of system justification and political orientation when studying the effect of the “meaning threat” posed by climate change. However, most studies are based on the American political system. To our knowledge, there are no studies addressing the specific link between environmental denial, system justification and political orientation in the French context and that is the second objective of this research.

## French political context

Although Jylhä and Akrami (2015) have shown that right political orientation in European context is associated with environmental denial and system justification, it is not clear how to draw a parallel with the French political system. In France, nearly a quarter of the population still doubts that global warming is occurring (Opinion Way Pour PrimesEnergie, 2019). Moreover, based on a recent national survey, Teinturier et al. (2019) showed that right political orientation (i.e., affiliation to “Rassemblement National” and “Les Républicains”) is descriptively associated with less concern for environmental issues. Similarly, Vasilopoulos and Lachat (2018) showed that right political orientation in France is positively associated with the concept of authoritarianism, which is also associated with system justification tendencies (Friesen et al., 2019). Taking into account these results, we hypothesized that the links established in the United States would be, in some way, similar in the French political system.

## Present research

With two studies, we address three main hypotheses. The first one is that when people are exposed to a threatening message that highlights the negative impacts of climate change for the French system, they will have a greater tendency to justify it and deny environmental problems (Study 1). The second hypothesis is that when people are exposed to a threatening message that highlights the growing pressure to change one’s habits, it would encourage them to deny environmental problems (Study 2). In both studies, we also expected that right political orientation will be associated with system justification tendencies and environmental denial. Data collection was undertaken between March and May 2019, before the COVID-19 pandemic. Data, materials and codes are available on the OSF repository.^1^ Both sample sizes were determined by time and resources constraints; we could only collect data from 150 students for each study. We justify the degree to which these samples are informative with sensitivity analyses. Also, incomplete data were not included in the final samples.

## Study 1

In the first study, we investigated how highlighting the threatening impacts of climate change for the French system could increase system justification tendencies and environmental denial while taking into account political orientation. To do so, we exposed undergraduate students to three types of video-clips (control vs. neutral vs. system threat) and we measured general system justification, environmental denial and political orientation. We expected that participants in system threat condition will have a greater score of system justification and environmental denial than those in control and neutral conditions. We also expected that a right political orientation will be positively associated with system justification and environmental denial.

### Method

#### Participants

One hundred and forty-eight undergraduate students in social sciences (114 females, 34 males, *M*_*age*_ = 20.45, *SD*_*age*_ = 2.54) were recruited on the campus in exchange for course credits. A power sensitivity analysis indicates that with this sample size, we would have been able to detect a minimal effect size (η^2^) of 0.077, given α = 0.05 and power (1–β) = 0.80.

#### Materials and procedure

The study was conducted at the university campus laboratory and was presented as a study on digital media communication methods. After signing the informed consent, the experimenter gave the instructions to the participant. At the end, all participants were debriefed.

To induce the environmental threat, three types of 1 min and 43 s video-clip were created (control vs. neutral vs. system threat). Videos of natural and human-made landscape videos were used, accompanied by a short text for the neutral vs. system threat conditions. A third control condition was necessary to avoid a possible effect of natural images presentation. Thus, in the control condition, participants were asked to watch the video with no text. In the neutral condition, participants watched the same video with a text about the force of gravity. In the system threat condition, the text highlighted threatening aspects of climate change, for example it contained sentences like “the French system will have to be completely restructured around climate change issues” and “France has a lot to learn and will soon be forced to change its system, its laws and its organization” (the complete texts are available on the Open Science Framework depository: see text footnote 1).

Environmental denial was measured with the 16 items (ω = 0.76) from Häkkinen and Akrami (2014) and general system justification was measured with the 8 items (ω = 0.84) from Kay and Jost (2003). Both scales were translated with a double-blinded approach. For political orientation, we asked participants to place themselves on a continuum from 1 (Extreme left orientation) to 9 (Extreme right orientation). Participants were mostly left-oriented (*M* = 3.97, *SD* = 1.28) and had rather low scores on system justification (*M* = 3.69, *SD* = 1.10) and on environmental denial (*M* = 2.27, *SD* = 0.78). All correlations are reported in Table 1.

**TABLE 1:** Intercorrelations for variables by study.

Variables	1	2	3
Political orientation	—	0.34***	0.24**
System justification	0.23**	—	0.27**
Environmental denial	0.24**	0.19	—

Correlations for study 1 (n = 148) are shown above the diagonal. Correlations for study 2 (n = 144) are shown below the diagonal. *p < 0.05. **p < 0.01. ***p < 0.001.

### Results

We analyzed our data with two multiple regression models with planned contrast codes for the type of video-clips, as recommended by Brauer and McClelland (2005). The first model tested the effect of the type of video-clips on system justification score while controlling for the interaction with political orientation. The second model tested the effect of the type of video-clips on the environmental denial score while controlling for the interaction with political orientation and also controlling for the system justification score. For each model, we tested both the main contrast code C1 (control = −1, neutral = −1, threat = + 2) and the residual contrast code C2 (control = −1, neutral = + 1, threat = 0).

The result for the first model indicated that there was no significant difference between the type of video-clips for C1, *b* = −0.19, 95% CI [−0.56, 0.19], *t*(142) = −0.97, *p* = 0.34, nor for C2, *b* = −0.07, 95% CI [−0.80, 0.67], *t*(142) = −0.18, *p* = 0.86. Thus, there was not enough evidence to suggest that system justification score was different between the control condition (*M* = 3.82, *SD* = 1.03) and neutral condition (*M* = 3.79, *SD* = 1.14) vs. the system threat condition (*M* = 3.50, *SD* = 1.14) (see Figure 1). However, the model confirmed that political orientation strongly and positively predicted system justification, *b* = 0.28, 95% CI [0.14, 0.41], *t*(142) = 4.04, *p* < 0.001, η_*p*_^2^ = 0.108. It means that the more people were right oriented, the more they justified their system. Although, political orientation did not appear to interact with the effect of threat on system justification, *b* = 0.03, 95% CI [−0.06, 0.12], *t*(142) = 0.61, *p* = 0.54, for the main contrast.

**FIGURE 1:** System justification score depending on video-clip type. Errors bars indicate the standard error.

The result for the second model indicated that the type of video-clips did not reach the significance level for both C1, *b* = 0.04, 95% CI [−0.23, 0.31], *t*(141) = 0.28, *p* = 0.78, and C2, *b* = 0.03, 95% CI [−0.50, 0.55], *t*(141) = 0.11, *p* = 0.91. Thus, there was not enough evidence to suggest that environmental denial score was different between the control condition (*M* = 2.20, *SD* = 0.77) and neutral condition (*M* = 2.48, *SD* = 0.84) vs. system threat condition (*M* = 2.17, *SD* = 0.73). As expected, system justification positively predicted environmental denial, *b* = 0.18, 95% CI [0.03, 0.27], *t*(141) = 2.49, *p* = 0.035, η_*p*_^2^ = 0.042, it means that higher system justification tendencies were associated with higher environmental denial score. Moreover, political orientation did not reach the significance level (although “marginally”), *b* = 0.10, 95% CI [−0.00, 0.20], *t*(141) = 1.97, *p* = 0.051, η_*p*_^2^ = 0.027, and, as the previous model, did not interact the effect of threat on environmental denial, *b* = −0.02, 95% CI [−0.08, 0.05], *t*(141) = −0.53, *p* = 0.60, for C1.

## Study 2

In the second study, we investigated how highlighting threatening aspects of climate change for individuals could increase environmental denial while taking into account the interaction with political orientation and also controlling for system justification tendencies. As study 1, we exposed undergraduate students to three types of video-clips (control vs. neutral vs. individual threat) and we measured system justification, environmental denial and political orientation. We expected that participants in threat condition will have a greater score of environmental denial than those in control and neutral conditions. We also expected that a right political orientation will positively predict environmental denial, controlling for system justification.

### Method

#### Participants

One hundred and forty-four undergraduate students in social sciences (111 females, 33 males, *M*_*age*_ = 20.65, *SD*_*age*_ = 2.50) were recruited on the university campus in exchange for course credits. With this sample size, we would have been able to detect a minimal effect size (η^2^) of 0.079, given α = 0.05 and power (1–β) = 0.80.

#### Materials and procedure

We used the same methodology as in study 1, participants were exposed to the same video-clips, except for the text accompanying the threat condition. In this study, we highlighted the necessity for individuals to change their way of life with sentences like “you will have to adopt a number of daily restrictions and eliminate your inappropriate behavior” or “You have a lot to learn and will soon be forced to change your habits and lifestyle” (the complete texts are available on the Open Science Framework depository: see text footnote 1).

Measures and scores were exactly the same as with study 1. Like the sample in study 1, participants were mostly left-oriented (*M* = 4.14, *SD* = 1.54) and had rather low scores for system justification (*M* = 3.60, *SD* = 1.09, ω = 0.76) and for environmental denial (*M* = 2.62, *SD* = 1.02, ω = 0.86). All correlations are reported in Table 1.

### Results

We conducted a multiple regression model with the same planned contrast codes used in study 1. We controlled for system justification and for the interaction between our conditions and political orientation.

For the type of video-clips, results did not reach the significance level for both the main contrast, *b* = −0.06, 95% CI [−0.35, 0.22], *t*(137) = −0.44, *p* = 0.659, and the residual contrast, *b* = 0.24, 95% CI [−0.24, 0.72], *t*(137) = 0.98, *p* = 0.330. Thus, the environmental denial score was not significantly higher in threat condition (*M* = 2.71, *SD* = 1.11) vs. control condition (*M* = 2.05, *SD* = 0.78) and neutral condition (*M* = 2.50, *SD* = 0.74) (see Figure 2). Moreover, system justification did not reach the significant level to predict environmental denial, *b* = 0.11, 95% CI [−0.03, 0.24], *t*(137) = 1.60, *p* = 0.112, η_*p*_^2^ = 0.018. The data also indicated that political orientation positively predicted environmental denial, *b* = 0.11, 95% CI [0.02, 0.20], *t*(137) = 2.30, *p* = 0.023, η_*p*_^2^ = 0.037. Thus, the more people declared themselves as right oriented, the more they presented high environmental denial scores. However, political orientation did not moderate the effect of threat on environmental denial, *b* = 0.05, 95% CI [−0.02, 0.12], *t*(137) = 1.52, *p* = 0.132, η_*p*_^2^ = 0.016, for the main contrast.

**FIGURE 2:** Environmental denial score depending on video-clip type. Errors bars indicate the standard error.

## General discussion

Our data did not support the hypotheses for system and individual threat but are consistent with the literature indicating that right political orientation and system justification are relevant factors when studying environmental denial. Thus, in both studies, the induction of environmental threat appears not to be effective. To discuss our failed manipulation, we propose three main explanations. First, our sample is mainly composed of young females, slightly left-oriented. Numerous articles have now demonstrated that system justification and threat responsiveness are stronger for men with a right-wing ideology (e.g., McCright and Dunlap, 2011). It is therefore possible that, because of the characteristics of our sample, we were not able to observe an effect of threat on system justification and environmental denial scores. Second, it is likely that our choice to induce environmental threat with texts in videos was not completely effective. Because we did not control for perceived threat between conditions, we cannot be sure that participants felt more or less threatened between conditions. A third explanation concerns our conceptualization of the environmental threat. While we distinguished two levels of this general meaning threat (i.e., system vs. individual), we did not focus on one specific consequence of climate change. It means that the content of the threatening messages may not have been specific enough. As a limitation, we are aware that the size of our samples may not have allowed us to detect the effect, if indeed it exists.

Moreover, the debate about the inconsistent effects of threatening messages on environmental attitudes is ongoing (e.g., Voelkel et al., 2021). While we find no evidence here to support the hypothesis that political orientation can moderate the effects of environmental threat, as proposed by Feygina et al. (2010), we contribute to this debate with additional data. Because “environmental threat” is composed of a wide range of threatening events, the definition of this threat and of political orientation may influence future hypotheses, specifically when researches are taking into account political ideologies (Crawford, 2017). One limitation is that, in these studies, we used a general environmental denial scale but it has recently been shown that studying specific forms of denial can lead to different outcomes (Wullenkord and Reese, 2021). It is all the more consistent that in the future, better use of denial forms will allow for better identification of psychological mechanisms in response to the environmental threat.

In addition, results are consistent with a considerable literature about the positive associations between right political orientation, system justification and environmental denial (e.g., Feygina et al., 2010; Häkkinen and Akrami, 2014). Thus, we found that a right political orientation is associated with higher tendencies to justify the system. This positive association contradicts recent results collected from a large sample of the French population (Langer et al., 2020) where authors found a negative association between political orientation and system justification tendencies (*r* = −0.17, *n* = 22 777). It indicates that people with left political orientation are more likely to justify their system than people with right political orientation. More recently, Vesper et al. (2022) find a positive, but non-significant correlation (*r* = 0.09, *n* = 463). One explanation is based on the nature of our sample, more precisely on the repartition of political orientation that is mostly centered and left oriented. Indeed, it is possible that our sample is more representative of young and left-oriented perceptions on the political spectrum. This implies that inter-individual differences that influence system justification tendencies should be understood as particularly dependent on the social, political and economic context.

## Conclusion

To conclude, although our data did not show an effect of environmental threat induction, they are consistent with previous associations found in the literature such as the positive link between right political orientation, system justification and environmental denial. This research contributes to both debates on the effects of environmental threat and on the role of political orientation to predict both system justification and environmental denial. It is therefore important to conduct more experimental studies on those questions, especially in different political contexts, and to use better definitions of environmental threat. One possibility is to investigate some political features that lead to the perception of threat from climate change messages. As Clarke et al. (2019) argued, a better definition of the threat will help to make better definitions and choice of outcomes. A good start would be to detail what is threatening, who will be threatened and when/where does it happen. Finally, we hope that this research can provide a first exploration of these issues in the French political context and that it can encourage people to investigate which aspects of climate change are perceived as threatening.

## Data Availability Statement

The original contributions presented in the study are publicly available. This data can be found here: https://osf.io/9k86r/.

## Ethics statement

Ethical review and approval was not required for the study on human participants in accordance with the local legislation and institutional requirements. The patients/participants provided their written informed consent to participate in this study.

## Author contributions

Both authors listed have made a substantial, direct, and intellectual contribution to the work, and approved it for publication.

## Conflict of Interest

The authors declare that the research was conducted in the absence of any commercial or financial relationships that could be construed as a potential conflict of interest.

## Publisher’s Note

All claims expressed in this article are solely those of the authors and do not necessarily represent those of their affiliated organizations, or those of the publisher, the editors and the reviewers. Any product that may be evaluated in this article, or claim that may be made by its manufacturer, is not guaranteed or endorsed by the publisher.

## Footnotes

1
https://osf.io/9k86r/
